The article "Tech Optimization in Cybersecurity Defenses by Advanced ML Methods: The Use Case of Volleyball Industry" was retracted in 2023. Reasons: signs of a paper mill; suspected computer-generated content; unreliable results or conclusions; concerns about the data.

# Tech Optimization in Cybersecurity Defenses by Advanced ML Methods: The Use Case of Volleyball Industry

**DOI:** 10.1155/2022/9907427

**Published:** 2022-05-17

**Authors:** Yuchun Xiao, Zhuo Bi, Zhibin Chen

**Affiliations:** ^1^Physical Education Teaching and Research Department, Hunan Institute of Technology, Hengyang 421002, China; ^2^Admissions and Career Service Office, Hunan Institute of Engineering, Xiangtan 411104, China

## Abstract

Individual and team performance can be improved by utilizing “smart” devices and applications that are connected through networks. In sports, the Internet of Things (IoT) refers to all of the “smart” devices and applications linked through networks to reduce injuries to the bare minimum, develop advanced training techniques, and apply analytical advanced sports improvement methodologies to improve sports performance in general. The Internet of Things (IoT) in sports is closely related to the objective of both security and privacy in sports, which has become a topic of crucial concern for the sports business in recent years, as evidenced by the adoption of IoT in sports years. For this reason, security flaws can have catastrophic consequences, including the disclosure of personal data, the manipulation of statistical findings, the harming of organizations' reputations, and enormous financial losses for the sporting organization. One or more of the consequences, as previously mentioned, is related to sports organizations and the athletes who are members of those organizations, and they have a direct impact on the corresponding set of sports-related, medical-related, and paramedical enterprises, specifically those that provide specialized sports equipment and associated services. A critical need to detect and quantify threats has long been recognized to better support decision-making when adopting or constructing a safe and reliable sports Internet-of-Things infrastructure, which is becoming increasingly common. Using advanced machine learning algorithms, this research provides a methodology for technology optimization in cybersecurity defenses that is then used in a unique case study utilizing volleyball players to demonstrate its effectiveness. In conjunction with a Monte Carlo optimization technique, an upgraded variant of fuzzy cognitive maps (FCM) is presented in greater detail. This model is utilized for a specific scenario of risk identification of volleyball industry, assessment, and optimization for IoT sports networks.

## 1. Introduction

The rapid development of modern sports technology contributes to increased performance and the impetus for exceeding the sport's limits. The big business giants of the sports industry invest in large-scale research for the development and production of state-of-the-art equipment products for athletes in collaboration with scientists, doctors, occupational physiologists, ergometers, and coaches [1]. The body of the athlete of each sport separately is simulated in special computer programs, where all the parameters that could potentially help produce a better athletic result are scientifically analyzed [2]. For these reasons, a set of wearable technologies sensors has been developed that are applied to countless links and fields of sports activity to assist in expanding human boundaries. These sensors are arranged in a sports IoT ecosystem, in which the bodies related to the sports industry participate [3].

Specifically, wearable athletic devices are small devices attached to the body in the form of a waistband or a skin patch. The gadgets then connect through Bluetooth and GPS, transmitting data in real time to IT equipment for analysis, recording, and feedback. Coaches and players can use data to improve performance, prevent injury, and reduce effort. For example, the impact monitor stickers alert coaches and trainers to possible concussions, brain trauma, overexertion, or injured muscles, tendons, and ligaments. Also, soft-tissue injuries can be identified early, allowing coaches to withdraw athletes before serious issues arise. GPS trackers sewed into the players' clothing track their balance, speed, acceleration, and mobility. In addition, IoT gadgets assess heart rate, metabolism, stress load, core temperature, and the physical repercussions of trauma.

However, the wide variety of “smart devices” in the sports industry introduces new security risks that make the industrial environment particularly dangerous in terms of cybersecurity. In a thorough effort to investigate the problem, the following causes are identified [4]:

1. Interconnected IoT devices mainly exchange “sensitive” data of athletes, which can be a pole of attraction for malicious activity and mainly black-market products.
2. Problems of complexity and incompatibility arise from the interaction of many devices and the heterogeneous networks that connect them.
3. As the IoT is a new and emerging sector, sports industry manufacturers are rushing to adopt smart system solutions without paying attention to security issues related to the confidentiality, integrity, and availability of the data and information they handle.
4. Most IoT sensors transmit and receive data wirelessly, and they carry the usual risks of wireless security breaches into the IoT sports ecosystem.
5. In addition, almost all IoT solutions include applications for their operation, monitoring, and control, the corresponding risks associated with software development and especially with authentication, authorization breaches, and the overall security and availability of these applications and connected databases.
6. The absence of solid computing resources in sports sensors is equivalent to the lack of strong encryption through “smart” sports devices, a fact that opens fields for the discovery and exploitation of the IoT network by malicious attackers.

Therefore, the pursuit of safety and privacy in sports IoT is a significant issue directly related to the evolution of the modern sports industry [5]. Based on the criticality of the environment in question in this work, a technique for optimizing cyber defense technologies using advanced machine learning methods is proposed. Specifically, a risk assessment model based on an advanced form of fuzzy cognitive maps (FCM) is presented [6], combined with a Monte Carlo optimization technique [7], which is applied to a specific scenario of risk identification, assessment, and optimization for the development of IoT sports networks.

## 2. Related Literature

The literature on cybersecurity and machine learning is rich, and the newer research focuses on dealing with the vast increase in cyber threats in modern information systems [8, 9].

Zhao et al. [10] looked at computational information approaches in IoT information security, such as computational intelligence-enabled cyberattacks and privacy services, cyber defense techniques, intrusion techniques, and data security. They also used computational intelligence capabilities to try to identify new study paths and trends for the growing IoT security challenges. They looked at the status of algorithmic intelligence-enabled cybersecurity concerns and IoT research trends. They outlined the primary obstacles that CI-enabled protection solutions face and new research topics that may be pursued. CI and cyber security-based strategies should be incorporated into the design of IoT to create robustness and make it more reliable.

Li [9] looked into two elements of the confluence of AI and digital protection. Deep learning may be used in cyber security to build intelligent models for malware categorization and intrusion detection. On the other side, AI models will be exposed to various cyberattacks, disrupting their sample, learning, and choices. To prevent adversarial machine learning, maintain privacy in machine learning, and safe federated training, AI models need cybersecurity and mitigation solutions. They then dissected the counterattacks that AI might face, categorized the appropriate defensive techniques, and examined the counterattacks that AI could face. Finally, they highlighted current research on developing a safe AI system from the standpoints of designing encrypted neural networks and implementing secure collaborative deep learning.

As the frequency of cyberattacks grows, Bresniker et al. [11] highlighted cybersecurity as a critical risk for every firm. Computational AI and machine training can assist cyber analysts in detecting threats and making suggestions and expanding the usage of AI/ML in cybersecurity needs worldwide collaboration between businesses, universities, and states. Companies are increasingly concerned about cyberattacks. Adequate cybersecurity necessitates automation, which requires recording cybersecurity analysts' actions. They believe that this will begin to happen soon, and because of the more significant usage of AI and ML in cybersecurity, assaults will become less successful and impactful.

Dasgupta et al. [12] conducted a review of recent work on machine learning in information security, describing the fundamentals of cyberattacks and their defenses, the fundamentals of the most frequently used methodologies, and suggested data mining strategies for information security in terms of capability, dimension reduction, and categorization techniques. This study also covers hostile machine learning and the security features of deep learning approaches. Finally, open topics, difficulties, and future research areas have been offered for aspiring researchers and engineers.

From the literature above, we conclude that researchers have identified that the sheer increase in cyberattacks can only be effectively dealt with the help of machine learning methodologies [12, 13].

## 3. FCM Methodology

The proposed implementation of technology optimization in cybersecurity defenses is based on the use of FCMs, which are a method of modeling complex systems capable of describing the causal relationships between critical factors' concepts that determine the behavior, symbolic description, and representation of system dynamics of cybersecurity used by the case study's sports organization [14].

FCMs are an excellent concept for analyzing the static and dynamic features of the IoT ecosystem and its evolving dynamic structure. Furthermore, it is an application motivated by various theoretical advancements recently revealed in IoT research. Moreover, the capacity of FCMs to forecast and classify time series is an intriguing element that aligns with the IoT specification.

In application view, FCMs provide concepts that describe various elements of system behavior and how these concepts are reacted to, either by their interaction or by the general dynamics of the system. Fuzzy rules are used to replicate the human experience and expertise of specialists who understand the function of system security and its behavior in various conditions. Each rule reflects an ideal situation or a specific system characteristic.

In our case, the designed FCM consists of nodes-concepts, *C*_*i*_, *i*=1,2,3,…, *N*, where *N* is the total number of ideas to be modeled systemically, which are its qualities, major factors, or properties. Concepts are linked together via connections with different weights, reflecting how concepts interact with one another [6].  Figure 1 depicts a basic concept of FCM.

In our example, there are three forms of causal links between two notions *C*_*i*_ and *C*_*j*_ [15]:

1. Positive: a positive weight indicates that an increase or reduction in the value of a causal concept leads this concept to move in the same direction *W*_*ij*_.
2. Negative: changes in the notions of cause and effect occur in opposite directions, as shown by the weight *W*_*ij*_ having a negative sign.
3. Nonexistent: It indicates an interconnection with zero weight. The value of weight, e.g., *W*_*ij*_, describes the concept *C*_*i*_ and affects the concept *C*_*j*_ and the interval [−1, 1].

At each time point, the value of each idea *A*_*i*_ is determined using a block function *f* from the sum of all the other concepts' influences and the total effect's limitation using the following rule [16]:

(1) $$\begin{array}{c} A_{i}^{t+1}=f\left(A_{i}^{t}+\sum_{i=1,\;i\neq j}W_{ji}A_{j}^{t}\right), \end{array}$$

where *A*_*i*_^*t*+1^ and *A*_*i*_^*t*^ are the concept's values *C*_*i*_ at time *t* + 1 and *t*, respectively, *A*_*j*_^*t*^  is the significance of the notion *C*_*j*_ at time *t*, *W*_*ji*_ is the connection's weight in the direction *C*_*j*_ to the meaning *C*_*i*_, and *f* is a block function that is used to limit the concept's value to a certain range, commonly in the interval [0, 1] [17, 18].

A new state of concepts emerges at each phase. After a specific number of repeats, the FCM can arrive at a point of equilibrium, a confined circle, or chaotic behavior. When the FCM reaches a given equilibrium point, it is concluded that the map has converged, and the end state corresponds to the real state of the system to which the values' transition when the map is applied.

The simulation activation function used calculates the value Α_*j*_ of a *C*_*j*_ concept at the end of an iteration as the sum of its causal concepts' contributions at the start of the iteration [6, 14, 18]:

(2) $$\begin{array}{c} A_{j}^{\left(t\right)}=f\left(\sum_{\begin{array}{c} i=1\\ i\neq j \end{array}}^{n}A_{i}^{\left(t-1\right)}w_{ij}+A_{j}^{\left(t-1\right)}\right), \end{array}$$

where *A*_*j*_^(*t*)^ is the value of the concept *C*_*j*_ at the end of the iteration, *A*_*i*_^(*t* − 1)^ is the value of the notation *C*_*j*_ at the beginning of the iteration, *w*_*ij*_ is the weight of the relation between *C*_*i*_ and *C*_*j*_, and *f* is a threshold function, which is used to normalize the values in each step. The process assumes that the weight table includes an autocorrelation by placing a unit value in the main diagonal of the table (the new value of the concept necessarily equals the previous value plus (or minus) the contribution of the other concepts associated with it). However, there is optional self-correlation because it is determined only by the values of the weight table's principal diagonal; as a result, self-correlation is implied and included in the first term of the equation, while the second term is ignored:

(3) $$\begin{array}{c} A_{j}^{\left(t\right)}=f\left(\sum_{i=1}^{n}A_{i}^{\left(t-1\right)}w_{ij}\right). \end{array}$$

In cases where there is no information about certain concepts/situations or experts/stakeholders cannot adequately describe the initial state of a variable, the equation takes the form:

(4) $$\begin{array}{c} A_{j}^{\left(t\right)}=f\left(\sum_{i=1}^{n}\left(2A_{i}^{\left(t-1\right)}-1\right)w_{ij}+2A_{j}^{\left(t-1\right)}-1\right). \end{array}$$

In case the problem incorporates the concept of time delay, the weight of a relationship with the value of the idea *I* at time *t* between recital node *i* and impact node *j* the lag_*ij*_ lag of the corresponding effect is

(5) $$\begin{array}{c} A_{j}^{\left(t\right)}=f\left(\sum_{\begin{array}{c} i=1\\ i\neq j \end{array}}^{n}A_{i}^{\left(t-{\text{lag}}_{ij}\right)}w_{ij}+A_{j}^{\left(t-1\right)}\right). \end{array}$$

The value of node *j* at time *t* is calculated as follows:

(6) $$\begin{array}{c} A_{j}\left(t_{n+1}\right)=f\left(\sum_{i=1}^{N}\mu_{ij}\left(t_{n}\right)\cdot A_{i}\left(t_{n}\right)\right), \end{array}$$

where *μ*_*ij*_(*t*_*n*_) is the value of the result of node *i* at node *j* at time *t*_*n*_. The value of the time function (*t*) depends on the type of function.

Finally, when the weights have not been defined before the start of the simulation but are dynamically adjusted during the simulation; the activation function for calculating the value of a concept has the following form:

(7) $$\begin{array}{c} A_{j}^{\left(t+1\right)}=A_{j}^{\left(t\right)}+\sum_{\begin{array}{c} i=1\\ i\neq j \end{array}}^{n}A_{i,\text{scaled }}^{\left(t\right)}w_{ij}. \end{array}$$

The above function is used to scale a value over an interval, as with the term *A*_*i*,scaled _^(*t*)^; the method does not use a threshold function [15, 18].

## 4. The Use Case of the Volleyball Industry

For the modeling of the proposed system, a specialized application scenario was implemented in the sports environment and specifically in a volleyball team. The usage scenario is based on optimizing the technological deployment cycle of IoT applications in cyber security. This particular sports volleyball team has several IoT technologies that do not make the most of their capabilities in the context of cyber security. The scenario aims to eliminate technology waste, make the most of already installed products, and maintain the responsibility of business application and information technology partners [13, 19].

The risk assessment process follows the steps below [20]:

1. Asset identification and prioritization: servers, customer contact information, critical partner documents, trade secrets, and other assets are examples of assets. Information on software, devices, features, data, interfaces, users, support, mission, purpose, operational needs, IT security policies, IT security architecture, network topology, data storage protection, information flow, and physical security environment is gathered for each component.
2. Threat identification: a threat could exploit a weakness to breach security and harm the team, including natural disasters, logical threats, and system failures' networks, inadvertent human interference, malicious acts, and vandalism.
3. Identifying vulnerability analysis: audit reports, vulnerability databases, incident response team data, and system software security analysis can all be used to identify vulnerabilities. Security and evaluation tests, penetration testing techniques, and automated vulnerability scanning are possible.
4. Controls' analysis: analyzing the controls in place or being designed reduces or eliminates the likelihood that a threat will exploit the system's vulnerability. Technical tools, such as hardware or software, encryption, intrusion detection measures, and authentication and authentication subsystems can be used to execute checks. Security policies, administrative activities, and physical and logical instruments are examples of nontechnical controls.
5. Calculating the likelihood of an event high, medium, and low categorization verbs examines the possibility of an assault or other adverse effects rather than numerical rating. The possibility of exploiting a vulnerability is calculated by considering the type of vulnerability, the ability and motive of the threat source, and the existence and efficacy of current measures.
6. Impact evaluation: a threat impact study considers the mission of the system, the methods it employs, its criticality, the value of the data handled, and the system's sensitivity.
7. Priority is given to information security risks: the level of risk to the system is determined for each threat/vulnerability pair based on the likelihood that the threat will exploit the vulnerability, the impact of successful exploitation of the exposure, and the adequacy of existing or planned security controls for the system to eliminate or reduce the risk.
8. Controls that are proposed: determine the steps to be made to mitigate the risk for each risk level using the risk level as a guideline: high, medium, and low.

The FCM's architecture is primarily reliant on the experience and expertise of a few experts, who, as experts, have enough knowledge to model a system and offer the initial values of the weights for the concepts' interconnections. In our situation, these weights are determined through a learning process [14]. The algorithm is iterated until a termination requirement, such as the maximum number of iterations or convergence to the target error based on a fitness metric is fulfilled. The FCM training algorithm is based on the Hebb rule and takes into account the fact that each node is activated asynchronously. This means that the balance of the map is accomplished by activating different nodes at different periods. As a result of this method, the FCM nodes are separated into activated nodes and nodes that will be activated. The node price renewal rule is adjusted in this scenario based on the following function [21, 22]:

(8) $$\begin{array}{c} A_{i}^{t+1}=f\left(A_{i}^{t}+\sum_{i=1,i\neq j}^{Ν}W_{ji}A_{j}^{\text{act}\left(t\right)}\right), \end{array}$$

where the act pointer indicates the activated node. The weight refresh rule based on this algorithm takes the form

(9) $$\begin{array}{c} w_{ij}^{\left(t+1\right)}=\left(1-\gamma^{\left(t\right)}\right)w_{ij}^{\left(t\right)}+\eta^{\left(t\right)}A_{i}^{\left(t\right)}\left(A_{j}^{\left(t\right)}-w_{ij}^{\left(t\right)}A_{i}^{\text{act}\left(t\right)}\right), \end{array}$$

where the learning rate *n* and the weight reduction factor in repetition *t* are calculated from the following equation:

(10) $$\begin{array}{c} \eta^{\left(t\right)}=b_{1}e^{\left(-\lambda_{1}t\right)},\gamma^{\left(t\right)}=b_{2}e^{\left(-\lambda_{2}t\right)}, \end{array}$$

where 0.01 < *b*_1_ < 0.09 and 0.1 < *λ*_1_ < 1, while *b*_2_ and *λ*_2_ are positive fixed numbers selected by test and observation.

The optimization problem based on the above modeling can be applied as a problem of finding the mean value and variance of the sum of random variables. Let 1 ≤ *i* ≤ *n* be random variables and *Z*=∑_*i*=1_^*n*^*X*_*i*_*i*. If *μx*_*i*_ = (*X*_*i*_) is the average value of 1 ≤ *i* ≤ *n*, then the mean value of Ζ is valid [23, 24]:

(11) $$\begin{array}{c} \mu_{Z}=E\left(Z\right)=E\left(\sum_{i=1}^{n}X_{i}\right)=\sum_{i=1}^{n}E\left(X_{i}\right). \end{array}$$

Let *Z* = *X* + *γ*, where *X* and *Y* are random variables. Then,

(12) $$\begin{array}{c} \sigma_{Z}^{2}=E\left[{\left(Z-\mu_{Z}\right)}^{2}\right]\Rightarrow \sigma_{Z}^{2}=E\left[{\left(X+Y-\mu_{X}-\mu_{Y}\right)}^{2}\right]\Rightarrow \\ \sigma_{Z}^{2}=E\left[{\left(X-\mu_{X}\right)}^{2}+2\left(X-\mu_{X}\right)\left(Y-\mu_{Y}\right)+{\left(Y-\mu_{Y}\right)}^{2}\right]\Rightarrow \\ \sigma_{Z}^{2}=E\left[{\left(X-\mu_{X}\right)}^{2}\right]+E\left[{\left(Y-\mu_{Y}\right)}^{2}\right]+2E\left[\left(X-\mu_{X}\right)\left(Y-\mu_{Y}\right)\right]. \end{array}$$

So, in the end, it turns out that the following relation holds for the variance:

(13) $$\begin{array}{c} \sigma_{Z}^{2}=\sigma_{X}^{2}+\sigma_{Y}^{2}+2\rho_{XY}\sigma_{X}\sigma_{Y}. \end{array}$$

The above relation is also generalized for the sum of *n* random variables:

(14) $$\begin{array}{c} \sigma_{z}^{2}=\sum_{i=1}^{n}\sigma_{i}^{2}+\sum_{i=1}^{n}\sum_{j=1\neq i}^{n}\sigma_{ij}, \end{array}$$

which is calculated as

(15) $$\begin{array}{c} \sigma_{z}^{2}=\left[\begin{array}{c} \sigma_{1}\sigma_{2}\sigma_{3}\cdots \sigma_{n} \end{array}\right]\cdot \left[\begin{array}{ccccc} 1 & \rho_{12} & \rho_{13} & \ldots & \rho_{1n}\\ \rho_{21} & 1 & \rho_{23} & \ldots & \rho_{2n}\\ \rho_{31} & \rho_{32} & 1 & \ldots & \rho_{3n}\\ \vdots & \vdots & \vdots & \ddots & \vdots \\ \rho_{n1} & \rho_{n2} & \rho_{n3} & \cdots & 1 \end{array}\right]\cdot \left[\begin{array}{c} \sigma_{1}\\ \sigma_{2}\\ \sigma_{3}\\ \vdots \\ \sigma_{n} \end{array}\right]=\sigma^{T}\cdot C\cdot \sigma . \end{array}$$

So, we use the collective risk model by looking at the IoT risks of the volleyball team with *X*_*ℏ*_ losses, the number of which is the random variable, as opposed to the individual risk model where we have a fixed number of losses. The random variables *X*_*h*_, ℏ = 1, 2,…, are losses and the random variable *N* is the number of losses that have occurred up to time *t*. Then, according to the collective risk model, the random variable of total losses is

(16) $$\begin{array}{c} S=\left\{\begin{array}{cc} X_{1}+X_{2}+\cdots +X_{N_{t}}, & N_{t}\geq 1,\\ 0, & N_{t}=0. \end{array}\right. \end{array}$$

To study the collective risk model, we assume that the random variables are independent. So, the moments of the random variable *S* for the collective risk model are given by the formulas:

(17) $$\begin{array}{c} E\left(S\right)=E\left(N_{t}\right)E\left(X\right),\\ \text{Var}\left(S\right)=E\left(N_{t}\right)\text{Var}\left(X\right)+\text{Var}\left(N_{t}\right)E^{2}\left(X\right). \end{array}$$

From the double mean theorem, we have

(18) $$\begin{array}{c} E\left(S\right)=E\left[E\left(S|N_{t}\right)\right]=E\left[E\left(X\right)N_{t}\right]=E\left(N_{t}\right)E\left(X\right), \end{array}$$

respectively, from the double mean theorem; for the variance, we have

(19) $$\begin{array}{c} \text{Var}\left(S\right)=E\left[\text{Var}\left(X\right)N_{t}\right]+\text{Var}\left[E\left(X\right)N_{t}\right]=\text{Var}\left(X\right)E\left(N_{t}\right)+E^{2}\left(X\right)\text{Var}\left(N_{t}\right). \end{array}$$

To find the distribution of the random variable and calculate the probability or probability density function, we use the convolution methodology. For the distribution function [25],

(20) $$\begin{array}{c} F_{S}\left(x\right)=\sum_{n=0}^{\infty }p_{n}F_{X}^{*}\left(x\right). \end{array}$$

And the proper tail function is

(21) $$\begin{array}{c} {\bar{F}}_{S}\left(x\right)=\sum_{n=1}^{\infty }p_{n}{\bar{F}}_{X}^{*}n\left(x\right). \end{array}$$

As we can conclude from the above example of risk modeling, with the distribution of individual and team risk assumed, the optimization process can prove to be highly beneficial for the optimal use of the sports IoT network studied. About the classical risk calculation and the independent application methodologies, the above methodology allows the application in a relatively easy, simple, and mainly automated way to change some of the application parameters of the system to create different equilibrium conditions and to re-evaluate the set of situations that affect the formation of risk about available existing-data, as well as to check the two-way interfaces under extreme cases.

## 5. Conclusions

The urgent need for intelligent detection and dynamic risk assessment in cases of instability, especially regarding cybersecurity, is an ongoing issue of concern to the research community. It is a severe and updated issue, especially when these risks are related to the support and decision-making processes when designing a safe and reliable sports IoT system. This study presents a methodology for tech optimization in cybersecurity defenses by advanced ML methods applied in a particular case study related to the volleyball industry. Specifically, a risk assessment model based on an advanced form of FCM is presented, combined with a unique form of Monte Carlo optimization, applied to a specific individual and collective risk scenario.

As proved, the proposed FCM is an excellent concept for assessing the IoT ecosystem's static and dynamic properties and its challenging structure as it evolves. Additionally, it is an application prompted by several recent theoretical breakthroughs in IoT research. FCMs give concepts that characterize various aspects of system behavior and how these concepts are reacted to, either through their interaction or through the system's overall dynamics. Fuzzy rules are used to emulate the human experience and skill of system security specialists who understand the function of the system and its behavior under varying conditions. Each rule is based on an ideal circumstance or a characteristic of a particular system.

A sophisticated application scenario is used to demonstrate the proposed multiscale simulation idea. This application aims to show how to apply the simulation concept, the core model, the building of detailed models, and the interpretation of simulation results. Because the simulation is relevant to all stages of production and diverse aims, the application displayed for IoT in sports is closely related to the purpose of security and privacy in sports, which has become a critical problem for the sports industry in recent years.

As a future research area, we suggest investigating more advanced optimization approaches, such as bio-inspired heuristic methods, that better reflect an IoT network's self-organization and development potential. Additionally, we believe that a hybrid methodology is necessary, in which the FCM may produce neural network topologies that can be deployed to any scenario-based solely on time limitations. Finally, some improvements must enhance the risk management process of cybersecurity defenses' methodologies, assessing and controlling potential threats.

## Figures and Tables

**Figure 1:** Simple FCM.

## Data Availability

The data used in this study are available from the author upon request.
